The article "Naloxone Protects against Lipopolysaccharide-Induced Neuroinflammation and Microglial Activation via Inhibiting ATP-Sensitive Potassium Channel" was published in 2021. Journal: Comput Math Methods Med.

# Naloxone Protects against Lipopolysaccharide-Induced Neuroinflammation and Microglial Activation via Inhibiting ATP-Sensitive Potassium Channel

**DOI:** 10.1155/2021/7731528

**Published:** 2021-07-29

**Authors:** Zhijia Tang, Xiaobao Shao, Jun Wu, Hucheng Chen, Anyu Zhang, Fei Xu, He Ping, Shiwei Li, Chunyan Liu, Yijun Li, Xue Xue, Binbin Yuan

**Affiliations:** ^1^Department of Medicine, Tongling Technology College, Anhui 244061, China; ^2^Department of Transfusion Medicine, The Affiliated Nanjing Traditional Chinese Medicine Hospital, Nanjing University of Chinese Medicine, Nanjing 210022, China; ^3^Department of Clinical Laboratory, Nanjing Brain Hospital & The Affiliated Brain Hospital of Nanjing Medical University, Nanjing 210029, China; ^4^Department of Nuclear Medicine, Nanjing First Hospital, Nanjing Medical University, Nanjing 210006, China; ^5^Department of Transfusion Medicine, Nanjing First Hospital, Nanjing Medical University, Nanjing 210006, China; ^6^Department of Neurosurgery, Haimen People's Hospital, Nantong 226100, China

## Abstract

**Aim:**

The aim of this study was to evaluate the anti-inflammatory effects and underlying mechanism of naloxone on lipopolysaccharide- (LPS-) induced neuronal inflammation and microglial activation.

**Methods:**

LPS-treated microglial BV-2 cells and mice were used to investigate the anti-inflammatory effects of naloxone.

**Results:**

The results showed that naloxone dose-dependently promoted cell proliferation in LPS-induced BV-2 cells, downregulated the expression of proinflammatory cytokines (TNF-*α*, IL-1*β*, and IL-6) and proinflammatory enzymes iNOS and COX-2 as well as the expression of free radical molecule NO, and reduced the expression of Iba-1-positive microglia in LPS-stimulated BV-2 cells and mouse brain. Moreover, naloxone improved LPS-induced behavior degeneration in mice. Mechanically, naloxone inhibited LPS-induced activation in the ATP-sensitive potassium (KATP) channel. However, the presence of glibenclamide (Glib), an antagonist of KATP channel, ameliorated the suppressive effects of naloxone on inflammation and microglial activation.

**Conclusion:**

Naloxone prevented LPS-induced neuroinflammation and microglial activation partially through the KATP channel. These findings might highlight the potential of naloxone in neuroinflammation therapy.

## 1. Introduction

Neuroinflammation, as a classic feature of neurodegenerative progression, has been observed in many diseases such as Alzheimer's disease, multiple sclerosis, and Parkinson's disease [1–3]. Substantial evidence has suggested that various cell types including neurons, astrocytes, and microglia are closely implicated in the process of neuroinflammation [4]. In particular, microglia, the major resident macrophages in the brain, play an important role in initial neuroinflammation [5]. Under pathological status, in response to detrimental stimuli, activated microglia could secret proinflammatory mediators such as tumor necrosis factor-*α* (TNF-*α*), interleukin-1*β* (IL-1*β*), and inducible nitric oxide synthase (iNOS) [6]. Overexpression of such proinflammatory factors could cause neuron damage which contributes to the development of neurodegenerative diseases [7]. Taking this into account, suppression of inflammation is considered beneficial for preventing neurodegenerative diseases.

Naloxone, a nonselective opioid receptor antagonist, has been known to possess potential anti-inflammation effects [8]. Structurally, naloxone has two stereoisomers, the (-) and (+) enantiomers. It has been documented that both isomers of naloxone can inhibit the release of inflammatory factors and microglial activation [9]. For instance, it has been suggested that naloxone could decrease the production of TNF-*α* and IL-1*β* and microglial activation induced by LPS in a model of Parkinson's disease [10]. Naloxone also reportedly blocks the inflammation process in endotoxin-activated murine macrophages [11]. Other study has shown that low concentration of naloxone could inhibit microglial activation and preserve the antinociceptive effect evoked by morphine in morphine-tolerant rats [12]. Despite evidence indicating the neuroprotective and microglial suppressive effects of naloxone, the underlying mechanisms by which it exerts the anti-inflammatory effects are complicated.

The expression of Kir6.1 increased significantly in the hypoxia-ischemia-reperfusion gerbil brain [13]. It was found that the SUR2 subunit was not necessary in mediating acute cardiovascular stress response; the level of SUR2 did not change obviously in the myocardial ischemia-reperfusion injury [14]. Moreover, it was reported that Kir6.2 and SUR2 were abundantly expressed in the nigral dopaminergic neurons and involved in the progress of neurological diseases [15, 16]. In the present study, the effects of naloxone on neuroinflammation and microglial activation induced by lipopolysaccharide (LPS) *in vitro* and *in vivo* were elucidated.

## 2. Materials and Methods

### 2.1. Cell Culture and Treatment

BV-2 microglial cells were purchased from the Chinese Academy of Science (Shanghai, China). Cells were cultured in Dulbecco's Modified Eagle Medium (DMEM) containing 10% fetal bovine serum (FBS) in a humidified atmosphere with 5% CO_2_ at 37°C. When cells grew to 80%-90% confluence, different concentrations of naloxone (0.5, 1.0, and 2.0 *μ*M) were added into the cells for 24 h in the presence or absence of LPS (1 *μ*g/mL) for 24 h.

### 2.2. CCK-8 Assay

BV-2 cells were cultured in 96-well plates at a density of 3 × 10^3^ cells/well. After 24 h, different concentrations of naloxone (0.5, 1.0, and 2.0 *μ*M) were added into cells for 48 h at 37°C followed by incubation with 10 *μ*L of CCK-8 reagents for another 4 h. At last, the absorbance was measured by a microplate reader.

### 2.3. Nitrite (NO) Detection

NO detection was performed using Griess's reagent kit (Invitrogen) according to the manufacturer's instructions. BV-2 cells were cultured and treated with different groups. The supernatant of the media was collected and mixed with the equal volume of Griess's reagent. The absorbance at the wavelength of 525 nm was measured by a microplate reader.

### 2.4. Animal Model

BALB/c mice (6-8 weeks, 20-22 g) were purchased from the Animal Laboratory of Nanjing University. Mice were fed in controlled conditions of temperature 25 ± 2°C, humidity 55%-65%, and 12 h light/dark cycle with free access to water and food. All the animal procedures were conducted in line with the Guidelines for Care and Use of Laboratory Animals of the University of Science and Technology of China and approved by the Animal Ethics Committee.

Mice were assigned into five groups: (I) control; (II) LPS—mice were intraperitoneally injected with LPS at a dose of 1.5 mg/kg on the last day and given saline as vehicle for 7 days; (III), (IV), and (V) LPS+naloxone—mice were administered naloxone (30 mg/kg, 60 mg/kg, and 90 mg/kg) for 7 days and injected with LPS on the last day. After 12 h of LPS treatment, mice were prepared for the behavior test. Finally, mice were sacrificed under anesthesia with 2% pentobarbital (50 mg/kg) for subsequent experiments as described with little modification [17]. After the rats were sacrificed, the brain was gently removed and postfixed in the same fixative (4% PF) overnight at 4°C. After dehydration, the brain tissues were embedded in paraffin and the serial paraffin-embedded 5 *μ*m thick sections were subjected to the subsequent analysis. For western blotting, the brains were immediately removed and frozen in liquid nitrogen and stored at -80°C until use.

### 2.5. Open Field Test

The behavioral changes were assessed by an open field test as described [18]. Briefly, mice were placed in a box (100 × 100 × 40 cm) and allowed to explore the area freely for 5 min. The activities were recorded by automatic software (Xinruan Information Technology, Shanghai, China). The movement parameters including number of rearings, distance traveled, and sitting time were quantified.

### 2.6. ELISA

Cells or brain tissues were collected for protein content quantification. The levels of TNF-*α*, IL-1*β*, and IL-6 were detected by ELISA kits (Beyotime, Shanghai, China) according to the manufacturer's directions.

### 2.7. Quantitative Real-Time Polymerase Chain Reaction (qRT-PCR)

Total RNA was extracted from cells using a TRIzol reagent (Invitrogen). 1 *μ*g of total RNA was inversely transcribed into cDNA. The expression levels of Kir6.2 and SUR2B were detected by qRT-PCR which was carried out by SYBR Premix EX Taq™. Relative gene expression was analyzed using the 2^-*ΔΔ*Cq^ method, and the levels were normalized to *β*-actin. The sequences for primes used were as follows: Kir6.2 forward: 5′-CGCATAAGAACATCCGTGAGC-3′, reverse: 5′-CAGCCACCACATGATAGCGAAG-3′; SUR2B forward: 5′-TTGACGATAGTACCCAGCTCCCT-3′, reverse: 5′-CAGATAATCCGTCCTGACCTCC-3′; and *β*-actin forward: 5′-TCCTTCCTGGGCATGGAGT-3′, reverse: 5′-CAGGAGGAGCAATGATCTTGAT-3′.

### 2.8. Western Blot

Total protein from cells or brain tissues was isolated using a radioimmunoprecipitation assay (RIPA) buffer (Beyotime, Shanghai, China), and the concentration was measured using a BCA kit (Beyotime, Shanghai, China). Protein was separated by a 12% SDS-PAGE gel and transferred to a PVDF membrane, followed by incubation with 5% nonfat milk in a Tris buffer at room temperature for 2 h. Afterwards, the membranes were incubated with primary antibodies at 4°C overnight. After washing with TBST for three times, the membranes were incubated with a goat anti-mouse HRP-conjugated IgG secondary antibody (1 : 5,000, ab97023, Abcam, Shanghai) for 2 h. Protein brands were visualized using an enhanced chemiluminescence kit (Beyotime, Shanghai, China). The primary antibodies used in this experiment were as follows: iNOS (1 : 250, ab15323), COX-2 (1 : 500, ab23672), Iba-1 (1 : 500, ab5076), *β*-actin (1 : 1,000, ab8227), Kir6.2 (1 : 500, ab251809), and SUR2B (1 : 1,000, ab84299). *β*-Actin was used as the internal control.

### 2.9. Immunofluorescence Assay

BV-2 cells were cultured in 6-well plates at a density of 1 × 10^5^ cells/well. After different treatments, cells were fixed in 4% paraformaldehyde and permeabilized with 0.2% Triton X-100 in PBS. Subsequently, cells were blocked and incubated with anti-Iba-1 antibody (ab5076) at 4°C overnight, followed by incubation with the related Alexa Fluor secondary antibody at room temperature for 2 h in the dark. At last, cells were stained with DAPI for 5 min. Images were acquired under a laser scanning confocal microscope (magnification, ×200).

### 2.10. Statistical Analysis

Data analysis was performed by using GraphPad Prism 5.0. Data was presented as mean ± standard deviation. One-way ANOVA analysis followed by Tukey's post hoc test was employed to compare differences between groups. A *P* < 0.05 was considered statistically significant.

## 3. Results

### 3.1. Naloxone Promoted LPS-Induced Cell Proliferation in BV-2 Cells

To investigate the effect of naloxone on cell viability of LPS-evoked BV-2 cells, cells were treated with different concentrations of naloxone in the presence or absence of LPS. The results of CCK-8 showed that naloxone had no significant effects on cellular proliferation of BV-2 cells (Figure 1(a)), indicating that naloxone at concentrations ranging from 0.5 to 2.0 *μ*M had no cytotoxicity on BV-2 cells. When challenged with 1 *μ*g/mL LPS for 24 h, BV-2 cells showed an obvious decrease in cell proliferation as compared to the control group (Figure 1(b)). Nevertheless, pretreatment with varying concentrations of naloxone for 24 h reversed the LPS-induced inhibitory effects on cell proliferation in a concentration-dependent manner. The outcomes suggested that naloxone had protective effects on the cellular proliferation of LPS-induced BV-2 cells.

### 3.2. Naloxone Attenuated LPS-Induced Inflammation and Microglial Activation in BV-2 Cells

It has been established that LPS usually triggers the release of inflammatory indicators from microglia [19]. Hence, whether naloxone had anti-inflammatory effects or not on LPS-stimulated BV-2 cells was studied. As an initial screening inflammatory indicator, NO has been reported to be involved in the process of microglia-mediated inflammation in the central nervous system (CNS) [20]. Firstly, the release of NO from BV-2 cells was examined. As shown in Figure 2(a), LPS treatment alone markedly promoted the release of NO compared with the control group, whereas incubation with naloxone before the addition of LPS mitigated the increase in NO levels triggered by LPS. Next, the levels of proinflammatory indicators were determined by ELISA. As revealed in Figures 2(b)–2(d), the levels of TNF-*α*, IL-1*β*, and IL-6 were dramatically elevated in LPS-exposed BV-2 cells compared to the control group. When treated with naloxone prior to LPS, the levels of TNF-*α*, IL-1*β*, and IL-6 were considerably repressed in a dose-dependent manner. In addition, naloxone pretreatment also caused a reduction in the protein expression of proinflammatory enzymes iNOS and COX-2, as evidenced by the results of western blot (Figure 2(e)). Collectively, these findings suggested that naloxone could eliminate LPS-stimulated inflammatory responses in BV-2 cells.

As the inherent immune cells of CNS, microglia could trigger neurodegenerative processes when activated [21]. To confirm the effects of naloxone on LPS-induced microglial activation in BV-2 cells, Iba-1 was used as a marker of microglia. The results of immunofluorescence staining showed that Iba-1-positive cells were increased in LPS-treated BV-2 cells, illustrating the activation of microglia (Figure 2(f)). However, microglial activation induced by LPS was significantly abolished by naloxone dose-dependently. These data identified that naloxone could suppress LPS-induced microglial activation in BV-2 cells.

### 3.3. Naloxone Improved LPS-Induced Behavioral Degeneration in Mice

Neuroinflammation has been shown to be correlated with behavior impairment [22]. To elucidate the locomotor activity of mice after LPS induction, an open field test was carried out. As depicted in Figure 3, it was found that LPS reduced the number of rearings and distance traveled and increased the sitting time in the box, as compared to the control group. More importantly, naloxone treatment dose-dependently increased the number of rearings and distance traveled and decreased the sitting time, as compared to the LPS-treated group, revealing that naloxone could alleviate the behavioral impairment caused by LPS.

### 3.4. Naloxone Suppressed LPS-Induced Inflammation and Microglial Activation in Mice

To figure out the roles of naloxone displayed in neuroinflammation and microglial activation inhibitory capacity *in vitro*, mice were treated with LPS to establish the neuroinflammation animal model. The results (Figure 4(a)) showed that the expression levels of proinflammatory cytokines (TNF-*α*, IL-1*β*, and IL-6) were dramatically accelerated after treatment with LPS but were significantly reduced after being incubated with naloxone, demonstrating the effective inhibitory properties of naloxone on the inflammation in mice. Moreover, consistent decrease was observed in the expressions of proinflammatory enzymes (iNOS and COX-2) after being treated with naloxone (Figure 4(b)). In addition, the western blot showed that LPS-induction contributed to the increase of Iba-1 expression, whereas naloxone restored it to a normal level in a dose-dependent manner (Figure 4(c)). It could be drawn from the findings that naloxone had protective effects on LPS-triggered neuroinflammation and microglial activation *in vivo*.

### 3.5. Naloxone Restrained LPS-Induced Activation of the KATP Channel *In Vitro* and *In Vivo*

The ATP-sensitive potassium (KATP) channel, expressed in excitable tissues like the brain, can directly modulate microglial activity and is a key ingredient of inflammatory responses following CNS injury [23, 24]. To figure out whether naloxone modulated the KATP channel, qRT-PCR and western blot were conducted to detect the expression levels of two subunits of the KATP channel (Kir6.2 and SUR2B). As depicted in Figures 5(a) and 5(b), the expression of Kir6.2 was notably upregulated in LPS-induced BV-2 cells compared with the control group, while the expression of Kir6.2 was distinctly reduced with the addition of naloxone in a concentration-dependent manner. Nevertheless, there was no obvious difference of naloxone on the expression of SUR2B in LPS-induced BV-2 cells. The expressions of Kir6.2 and SUR2B in the LPS-treated mouse brain clearly exhibited the similar extension with the administration of naloxone (Figures 5(c) and 5(d)). Altogether, the above data proved that naloxone potentially exhibited a suppressive regulation on the KATP channel.

### 3.6. Naloxone Protected LPS-Induced Neuroinflammation and Microglial Activation via Inhibiting the KATP Channel

To gain insights into the mechanism involved in the inhibitory effects of naloxone on LPS-stimulated inflammation, glibenclamide (Glib), an antagonist of the KATP channel, was used to validate the changes in LPS-associated neuroinflammation and microglial activation. Firstly, cells were pretreated with Glib (10 *μ*M) for 1 h before being subjected to LPS stimulation and naloxone treatment. Then, a CCK-8 assay was performed. As a consequence, pretreatment with Glib distinctly reversed the protective role of naloxone on cell proliferation in LPS-induced BV-2 cells (Figure 6(a)). To find out whether the KATP channel was involved in the inflammatory response, ELISA, NO analysis, and western blot were conducted to measure the release of proinflammatory cytokines in the presence of Glib. As expected, the naloxone-induced decrease of NO, TNF-*α*, IL-1*β*, IL-6, iNOS, and COX-2 in LPS-treated BV-2 cells was markedly neutralized by Glib (Figures 6(b)–6(d)). Similar to the above data, KATP channel inhibition using Glib pronouncedly counteracted the regulatory effect of naloxone on microglial activation in BV-2 cells cocultured with LPS (Figure 6(e)). Jointly, these results revealed that the protective effects of naloxone on neuroinflammation and microglial activation in LPS-induced BV-2 cells could be diminished by the suppression of the KATP channel.

## 4. Discussion

In this study, the neuroinflammation-protective effects and mechanisms of naloxone were characterized in LPS-stimulated BV-2 cells and mice. The findings suggested that naloxone prevented the neuroinflammation by decreasing the release of inflammatory mediators including NO, TNF-*α*, IL-1*β*, and IL-6 as well as the expression of iNOS and COX-2 in a dose-dependent manner. Naloxone also reduced the expression of Iba-1, a key indicator of microglial activation. In addition, naloxone was found to improve the behavior impairments triggered by LPS in mice. Finally, utilizing the inhibitor of the KATP channel, naloxone was verified to exert the protective effects of neuroinflammation and microglial activation via the KATP channel.

It is commonly known that inflammatory response is a major factor to the development of neurodegeneration [25]. To mimic the inflammatory response, LPS was used as an inflammatory activator [26]. Following LPS exposure, the overexpression of TNF-*α*, IL-1*β*, and IL-6 was observed, which was consistent with the previous study that LPS triggered the release of proinflammatory cytokines [27–29]. However, naloxone decreased the levels of these proinflammatory cytokines in a dose-dependent manner. Importantly, COX-2 has been reported to be implicated in proinflammatory stimuli such as TNF-*α*, IL-1*β*, and IL-6 [30]. NO, produced by iNOS, plays an important regulatory role in homoeostasis, but it may be pathogenic when generated excessively [31]. This study showed the increased expression of iNOS, COX-2, and NO after LPS induction; naloxone was found to alleviate the production of these mediators. Taken together, these findings indicated that naloxone had considerable neuroprotective effects on LPS-induced inflammation, which agreed with the findings of published researches [12, 32]. The results of the CCK-8 assay also confirmed that naloxone exerted a cellular protective effect in neuroinflammation damage.

Microglia, as the frontier line of immune defense in CNS, play a crucial role in response to injury and pathogens. Sustained activation of microglia is involved in the progress of neurodegenerative diseases. Suppression of microglial activation has been demonstrated to protect against neurodegenerative changes [33]. Naloxone has been reported to exert a neuroprotective effect through inhibiting microglial activation in models of light-triggered photoreceptor degeneration [34]. Naloxone effectively prevented microglial activation in LPS-induced retinal cells [35]. In the current study, it was found that LPS treatment activated microglia, while naloxone effectively restrained the microglial activation dose-dependently, which was consistent with existing publications. Moreover, activated microglia usually release abundant proinflammatory cytokines, which was supported by the above results of proinflammatory indicators.

The ATP-sensitive potassium (KATP) channel is in different encephalic regions with different types of subunits including Kir6.1, Kir6.2, SUR1, and SUR2. In line with the current study, multiple studies verified that the inhibition of the KATP channel exhibited a neuroprotective effect. For instance, blockade of the KATP channel protected neurons against neurodegenerative stimuli [36]. This study further showed that the KATP blocker Glib mitigated the protective effects of naloxone against LPS-induced neuroinflammation in BV-2 cells, indicating that the protective effects of naloxone on neuroinflammation were partly through the KATP channel. Given that the macrophage NLRP3 inflammasome activation is inhibited by potassium channel inhibition [37], inhibiting the ATP-sensitive potassium channel is not the only main reason for explaining the underlying anti-inflammatory mechanism of naloxone. We are exploring the detailed inflammasome activation pathway and its close relationship with the ATP-sensitive potassium channel in this model.

In summary, this study demonstrated that naloxone inhibited neuroinflammation and microglial activation in LPS-induced BV-2 cells and the mouse brain. Moreover, the data provided evidence for the neuroinflammation-protective effects of naloxone via inhibition of the KATP channel based on the *in vitro* and *in vivo* study.

## Figures and Tables

**Figure 1:** Effects of naloxone on the cell proliferation of BV-2 cells. (a) The effect of naloxone on the cell proliferation was detected by CCK-8. (b) The effect of naloxone on the cell proliferation in LPS-induced cells was detected by CCK-8. ^∗^*P* < 0.05.

**Figure 2:** Effects of naloxone on the inflammatory responses and microglial activation in LPS-induced BV-2 cells. (a) The release of NO was measured by Griess's kit. (b–d) The expressions of proinflammatory cytokines TNF-*α*, IL-1*β*, and IL-6 were measured by ELISA. (e) The expressions of proinflammatory enzymes iNOS and COX-2 were determined by western blot. (f) The expression of Iba-1 in LPS-induced BV-2 cells was evaluated by immunofluoresence. ^∗^*P* < 0.05; ^∗∗^*P* < 0.01.

**Figure 3:** Effect of naloxone on the behavior impairment induced by LPS in mice was assessed by open field test. ^∗^*P* < 0.05; ^∗∗^*P* < 0.01.

**Figure 4:** Effects of naloxone on the inflammatory response and microglial activation induced by LPS *in vivo*. (a) The expressions of proinflammatory cytokines TNF-*α*, IL-1*β*, and IL-6 were measured by ELISA. (b) The expressions of proinflammatory enzymes iNOS and COX-2 were determined by western blot. (c) Effect of naloxone on the expression of Iba-1 in mouse brain was determined by western blot. ^∗^*P* < 0.05; ^∗∗^*P* < 0.01.

**Figure 5:** Effects of naloxone on the expressions of KATP channel. (a) The mRNA expressions of Kir6.2 and SUR2B in LPS-stimulated BV-2 cells were examined by qRT-PCR. (b) The protein expressions of Kir6.2 and SUR2B in LPS-stimulated BV-2 cells were examined by western blot. (c) The mRNA expressions of Kir6.2 and SUR2B in LPS-stimulated mouse brain were examined by qRT-PCR. (d) The protein expressions of Kir6.2 and SUR2B in LPS-stimulated mouse brain were examined by western blot. ^∗^*P* < 0.05.

**Figure 6:** Naloxone exerted protective effects of neuroinflammation induced by LPS through KATP channel. (a) The effect of naloxone on the cell proliferation in LPS-induced cells was detected by CCK-8. (b) The expressions of proinflammatory cytokines TNF-*α*, IL-1*β*, and IL-6 were measured by ELISA. (c) The release of NO was measured by Griess's kit. (d) The expressions of proinflammatory enzymes iNOS and COX-2 were determined by western blot. (e) The effect of naloxone on the expression of Iba-1-positive cells was evaluated by immunofluoresence. ^∗^*P* < 0.05; ^∗∗^*P* < 0.01.

## Data Availability

All data generated or analyzed during this study are included in this published article.
